# The clinical prognostic significance of ezrin in patients with bone and soft tissue sarcomas: a meta‐analysis

**DOI:** 10.1002/2211-5463.12713

**Published:** 2019-09-03

**Authors:** Feng Wang, Tao Yu, Chengbin Ma, Haifei Zhang, Zhiyu Zhang

**Affiliations:** ^1^ Department of Orthopedics the Fourth Affiliated Hospital of China Medical University Shenyang Liaoning China; ^2^ Center for Translational Medicine the Fourth Affiliated Hospital of China Medical University Shenyang Liaoning China

**Keywords:** ezrin, meta‐analysis, overall survival, prognosis, sarcoma

## Abstract

Ezrin is a member of the ezrin–radixin–moesin (ERM) protein family and has been shown to be associated with poor prognosis in patients with a variety of solid tumors. However, the clinical prognostic significance of ezrin in patients with bone and soft tissue sarcomas remains unclear. Here, we performed a systematic meta‐analysis by searching PubMed, the Cochrane Library Database, EMBASE, the Web of Science, and the CBM, WanFang Med Online and CNKI databases. In total, 19 studies with a total of 1316 bone and soft tissue sarcoma patients were included. Pooled analyses showed that ezrin overexpression was correlated with a higher rate of tumor metastasis (OR 6.59, 95% CI: 2.84–15.33, *P* < 0.01, *P*_FDR_ < 0.01) and recurrence (OR 3.18, 95% CI: 1.88–5.37, *P* < 0.01, *P*_FDR_ < 0.01) and a more advanced tumor grade (OR 3.252, 95% CI: 1.371–7.715, *P* = 0.01, *P*_FDR_ = 0.03). Moreover, elevated ezrin expression could predict poor OS (HR 3.02, 95% CI: 2.35–3.89, *P* < 0.01, *P*_FDR_ < 0.01), MFS (HR 5.22, 95% CI: 2.08–13.08, *P* < 0.01, *P*_FDR_ < 0.01), and EFS (HR 1.07, 95% CI: 1.03–1.11, *P* < 0.01, *P*_FDR_ < 0.01). Subgroup analyses revealed the underlying sources of heterogeneity. Publication bias was observed in the analysis of metastasis. Sensitivity analysis revealed that the results were robust. Our findings indicated that ezrin overexpression was significantly correlated with poor survival and more advanced tumor progression in bone and soft tissue sarcomas, which suggests that ezrin might be a valuable prognostic biomarker and a potential therapeutic target.

**Abbreviations**
CI: confidence interval
DSS: disease‐specific survival
EFS: event‐free survival
ERM: ezrin–radixin–moesin
FDR: false discovery rate
HR: hazard ratio
IHC: immunohistochemistry
MFH: malignant fibrous histiocytoma
MFS: metastasis‐free survival
NOS: Newcastle–Ottawa Scale
OR: odds ratio
OS: overall survival
STS: soft tissue sarcoma
TMA: tissue microarray

Bone and soft tissue sarcomas are a group of malignancies that originate from mesenchymal tissues and are classified as either primary bone sarcoma or soft tissue sarcoma. Advances in their treatment have improved the survival rate of patients with bone and soft tissue sarcoma 1, 2, 3. However, patients with high‐grade sarcomas or the metastasis/recurrence of disease still suffer a great deal, and their survival rates are low 4. In addition to surgical and chemo/radio‐therapeutic interventions for patients with bone and soft tissue sarcomas, the molecular and genetic mechanisms of bone and soft tissue sarcomas have been widely investigated to identify a number of molecular biomarkers that could be used to predict the prognosis of patients with bone and soft tissue sarcomas 5, 6, 7, 8. However, bone and soft tissue sarcomas have high heterogeneity, and the outcomes are limited. Further investigation is needed to explore potential biomarker(s) that might be used to predict the prognosis of patients with bone and soft tissue sarcomas.

Ezrin is a member of the ezrin–radixin–moesin (ERM) protein family, which is highly evolutionarily conserved and essential for many cellular processes, such as the formation of cytoskeletal linkers. In cancer progression, ezrin is involved in cell adhesion, migration, and invasion as well as tumor growth and metastasis by acting as a key molecule involved in membrane organization or cellular signal transduction 9, 10, 11, 12. Due to the potential importance of ezrin in cancer, the prognostic significance of ezrin has been evaluated in numerous types of cancers 13, 14, 15, 16. However, the results have been somewhat contradictory 15, 17, 18. Recent meta‐analyses have revealed that elevated ezrin expression is associated with poor prognosis in patients with a variety of solid tumors 19, 20. However, the prognostic and clinicopathological significance of ezrin in patients with bone and soft tissue sarcomas remains unclear.

In the present meta‐analysis, the correlations between ezrin expression and prognostic and clinicopathological outcomes (CP) were evaluated to investigate whether ezrin expression could serve as a prognostic and clinicopathological biomarker for patients with bone and soft tissue sarcomas.

## Materials and methods

### Search strategies

There were seven databases in total that were used to comprehensively search the electronic publications for the meta‐analysis: PubMed, the Cochrane Library Database, EMBASE, the Web of Science, and the CBM, WanFang Med Online and CNKI databases. The search was updated in June 2018, and no restrictions in terms of language or publication date were used; the last search was conducted on June 30, 2018. The search terms used for the meta‐analysis were as follows: ‘ezrin’ or ‘cytovillin’ or ‘villin 2’ and ‘sarcoma’ or ‘soft tissue sarcoma (STS)’ or ‘bone sarcoma’ or ‘osteosarcoma’ or ‘chondrosarcoma’ or ‘Ewing sarcoma’ or ‘leiomyosarcoma’ or ‘angiosarcoma’ or ‘malignant fibrous histiocytoma (MFH)’ or ‘liposarcoma’ or ‘rhabdomyosarcoma’ or ‘synovial sarcoma’. Moreover, the reference lists in each of the identified studies were manually searched to avoid missing potentially relevant studies.

### Inclusion and exclusion criteria

The following criteria were employed to include eligible studies in the meta‐analysis: (a) addressed patients with pathologically confirmed bone and soft tissue sarcomas; (b) focused on the correlations between ezrin expression and the clinicopathological and prognostic outcomes of patients with bone and soft tissue sarcoma; (c) provided odds ratios (ORs) and/or hazard ratios (HRs) along with the 95% confidence intervals (CIs) or data that could be used to estimate these statistics; and (d) utilized defined cutoff values to classify ezrin expression as ‘positive’ and ‘negative’ or ‘high’ and ‘low’ or provided data that could be used to classify ezrin expression as ‘positive’ and ‘negative’ or ‘high’ and ‘low’ according to a given classification. Studies were excluded if they (a) were reviews, letters, case reports, or conference abstracts; (b) involved nonhuman research, including animal experiments and cell experiments; (c) were not related to ezrin expression; (d) used a small sample size if the reported data were overlapping; and (e) contained insufficient data to allow the estimation of the statistics of related outcomes and had sample size less than 30. Two authors independently determined the eligibility of the included studies. Any discrepancy was resolved by consensus after discussion.

### Data extraction and quality assessment

The data of interest were extracted independently by two authors and included the following information: (a) basic characteristics (first author, publication year, sample size, language, tumor type, patient source, use of prechemotherapy/radiotherapy, presence of positive ezrin expression, testing method, subcellular location of ezrin staining, and the cutoff value); (b) HRs for survival outcomes, including overall survival (OS), metastasis‐free survival (MFS), and event‐free survival (EFS)/disease‐specific survival (DSS), and the relevant 95% CIs, which were extracted directly from the study or estimated according to Tierney’s method 21; and (c) data that could be used to estimate the ORs for the correlations between ezrin expression and CPs. When HRs obtained from both univariate and multivariate analyses were available, the HRs from the multivariate analysis were used.

The methodological quality of each study was assessed by using the Newcastle–Ottawa Scale (NOS) (www.ohri.ca/programs/clinical_epidemiology/oxford.asp) system. There are three quality parameters in the NOS tool: selection (0–4 stars), comparability (0–2 stars), and outcome assessment (0–3 stars). One star was awarded when a study met the requirements of each item, and studies with an NOS score ≥ 6 stars were considered to be of high quality and included in the meta‐analysis.

### Statistical analysis

The HRs and ORs, as well as their 95% CIs, were used to assess the pooled prognostic and clinicopathological significance of ezrin expression. A HR < 1 suggested a more favorable prognosis, and a HR > 1 suggested a worse prognosis in sarcoma patients. An OR > 1 indicated a positive correlation between ezrin expression and CPs. Chi‐square tests and *I* ^2^ tests were used to analyze the interstudy statistical heterogeneity. When there was no significant heterogeneity (*P *> 0.10 or *I* ^2^ < 50%), a fixed‐effects model was appropriately used to calculate the pooled effect; otherwise, a random‐effects model was used. If there was obvious heterogeneity, a subgroup meta‐analysis was conducted to identify the underlying heterogeneity. Moreover, a funnel plot analysis, Begg's tests, and Egger's tests were used to assess the publication bias. If there was an obvious publication bias, a trim‐and‐fill analysis was used to determine the underlying origin of the publication bias. A sensitivity analysis was used to assess the stability of the pooled results when at least five studies were included. To control for the proportion of false positives, the Benjamini–Hochberg method of determining the false discovery rate (FDR) was applied to adjust the *P* value, and *P* < 0.05 was considered statistically significant. All analyses were performed by using stata version 14.0 (Stata Corporation, College Station, TX, USA).

## Results

### Study selection

A total of 351 studies were identified initially using our strategy for a comprehensive search of PubMed, the Cochrane Library Database, EMBASE, the Web of Science, and the CBM, WanFang Med Online and CNKI databases. After discarding duplicates, 153 studies were subject to further screening. After title and abstract screening, 96 studies were excluded. Out of 57 studies, 33 studies were omitted due to irrelevance. For further eligibility evaluation, the full‐text articles were read, and five studies were removed because of overlapping data (*n* = 2) and insufficient data (*n* = 3). Therefore, 19 studies 17, 22, 23, 24, 25, 26, 27, 28, 29, 30, 31, 32, 33, 34, 35, 36, 37, 38, 39 with 1316 bone and soft tissue sarcoma patients were included in the meta‐analysis, and data from 13 studies were used to evaluate the clinicopathological significance and data from 17 studies were used to evaluate the prognostic value of ezrin expression. A flow diagram of the selection process is shown in Fig. 1.

**Figure 1:** Flow diagram of the study selection process.

### Characteristics and quality assessment of the eligible studies

The summarized study characteristics and the quality assessment are shown in Table 1. Briefly, the studies included were written either in English (*n* = 13) or in Chinese (*n* = 6). The patients were collected internationally from Asian (*n* = 10) and non‐Asian (*n* = 9) populations. The sample size ranged from 34 to 227 with a median of 57. Six types of bone and soft tissue sarcomas were investigated in the studies: osteosarcoma (*n* = 12), Ewing sarcoma (*n* = 1), synovial sarcoma (*n* = 1), STS (*n* = 3), myxofibrosarcomas (*n* = 1), and MFH (*n* = 1). Immunohistochemistry (IHC) was employed to evaluate ezrin expression in all of the studies. Ezrin expression was defined as staining in the cytoplasm and/or membrane, and cutoff values were available for all studies. Moreover, data from 13 studies, four studies, and five studies were extracted to analyze the HRs of OS, MFS, and EFS/DSS, respectively. Using the NOS tool, the quality of each study included was assessed, and all of the studies were found to be of high quality, with scores ranging from 6 stars to 9 stars.

**Table 1:** Characteristics and quality assessment of the included studies. C, cytoplasm; M, membrane; NR, not reported; STS, soft tissue sarcomas.

Study	Year	Sample size (*n*)	Language	Tumor type	Source	Pretherapy (Y/N)	Positive (high)/negative (low)	Staining method	Staining position	Cutoff value	Prognostic value	Clinical value	NOS
Cash T	2017	53	English	Ewing sarcoma	USA	Y	38/15	IHC	C/M	≥ 1% of cells	EFS	CP	9
Abdou AG	2016	57	English	Osteosarcoma	Egypt	N	47/10	IHC	C/M	> 0% of cells	‐	CP	7
Ni Z	2016	44	Chinese	Osteosarcoma	China	Y	21/23	IHC	C	Score ≥ 2	OS	CP	7
Tang ZB	2016	58	Chinese	Osteosarcoma	China	Y	34/24	IHC	C	Score ≥ 2	OS	CP	8
Palmerini E	2015	88	English	Synovial sarcoma	Italy	Y/N	80/8	IHC	C/M	> 0% of cells	OS	‐	9
Xilin BLR	2015	94	Chinese	STS	China	Y/N	44/50	IHC	M	Score ≥ 4	‐	CP	8
Le Guellec S	2013	35	English	Osteosarcoma	France	Y	11/24	IHC	C	Score > 6	OS, MFS	‐	8
Min DL	2012	82	Chinese	Osteosarcoma	China	N	49/33	IHC	C	Score ≥ 1	OS	CP	6
Carneiro A	2011	227	English	STS	Sweden	Y/N	154/73	TMA‐IHC	C/M	Score ≥ 4	MFS	CP	8
Boldrini E	2010	34	English	Osteosarcoma	Brazil	N	26/8	IHC	C/M	> 0% of cells	OS	‐	8
Huang HY	2010	74	English	Myxofibrosarcomas	Taiwan	NR	35/39	TMA‐IHC	C/M	≥ 50% of cells	MFS, DSS	CP	8
Yang JZ	2010	51	Chinese	Osteosarcoma	China	Y	20/31	IHC	C	> 0% of cells	OS	CP	6
Kim C	2009	70	English	Osteosarcoma	Korea	Y	39/31	IHC	C	≥ 10%	OS, EFS	CP	8
Shen XD	2008	56	Chinese	Osteosarcoma	China	Y	38/18	TMA‐IHC	C	> 0% of cells	OS	CP	9
Ferrari S	2008	95	English	Osteosarcoma	Italy	Y	76/19	IHC	C/M	≥ 1% of cells	EFS	CP	7
Kim MS^a^	2007	47	English	MFH	Korea	Y/N	27/20	TMA‐IHC	C/M	≥ 10% of cells	OS, MFS	CP	9
Kim MS	2007	64	English	Osteosarcoma	Korea	N	33/21	IHC	C	> 0% of cells	OS, MFS	CP	7
Salas S	2007	37	English	Osteosarcoma	France	Y	23/14	IHC	C/M	≥ 1% of cells	OS, EFS	CP	8
Weng WH	2005	50	English	STS	Sweden	N	25/25	IHC	C/M	≥ 1% of cells	OS	CP	8

### Correlation between ezrin expression and survival outcomes

As no obvious heterogeneity was observed in the analysis of OS (*I* ^2^ = 22.40%, *P* = 0.22) and EFS (*I* ^2^ = 38.90%, *P* = 0.18), a fixed‐effects model was used for each analysis. A random‐effects model was used for the analysis of MFS (*I* ^2^ = 78.30%, *P* = 0.00). The pooled overall effects (Fig. 2) showed that elevated ezrin expression was correlated with poor OS (HR 3.02, 95% CI: 2.35–3.89, *P* < 0.01, *P*_FDR_ < 0.01; Fig. 2A), MFS (HR 5.22, 95% CI: 2.08–13.08, *P* < 0.01, *P*_FDR_ < 0.01; Fig. 2B), and EFS (HR 1.07, 95% CI: 1.03–1.11, *P* < 0.01, *P*_FDR_ < 0.01; Fig. 2C). For the analysis of DSS, original data were extracted from only one study 26 and indicated that elevated ezrin expression could predict poor DSS (HR 4.54, 95% CI: 2.92–40.89, *P* = 0.03; Table 2); however, after FDR adjustment, no statistical significance was observed (*P*_FDR_ = 0.09). As most of the extracted data were obtained from patients with osteosarcoma, and in order to evaluate if the prognostic value of ezrin expression was limited to osteosarcoma, in the analysis of OS and EFS, a subgroup analysis according to tumor type (osteosarcoma vs. nonosteosarcoma) was performed. The results showed that ezrin overexpression could predict poor OS in both osteosarcoma (HR 3.15, 95% CI: 2.39–4.14, *P* < 0.01, *P*_FDR_ < 0.01) and nonosteosarcoma (HR 2.38, 95% CI: 1.24–4.58, *P* = 0.01, *P*_FDR_ = 0.01). However, ezrin overexpression failed to predict poor EFS in osteosarcoma (HR 1.20, 95% CI: 0.74–1.96, *P* = 0.46, *P*_FDR_ = 1.38, random‐effects; Table 2), which might have been caused by the limited number studies used and indicates the presence of obvious heterogeneity. In the analysis of MFS, stratified analyses according to sample size and source, analysis model, publication date, and tumor type were conducted to investigate the underlying source of heterogeneity. The results showed that sample size and source and publication date might be sources of underlying heterogeneity, and the prognostic value of ezrin expression was not altered (Table 2). As chemo/radiotherapy was of great importance to the prognosis of sarcoma patients, a stratified meta‐analysis according to the use of pretherapy (Y/N) was conducted in the analysis of OS. In total, 11 studies were included, and no obvious heterogeneity in the meta‐analysis was observed (*I* ^2^ = 26.9%, *P* = 0.19, fixed‐effects). Ezrin overexpression was correlated with poor OS, regardless of whether the patients received chemo/radiotherapy (HR 2.96, 95% CI: 2.28–3.84, *P* < 0.01, *P*_FDR_ < 0.01) before surgery, as shown in Table 2.

**Figure 2:** Forest plots of pooled HR for OS (A), MFS (B), and EFS (C).

**Table 2:** Summary of correlation between ezrin expression and survival outcomes.

Subgroup	Study (*n*)	HR (95% CI)	*P*	*P*_FDR_	Heterogeneity	
					*I* ^2^ (%)	*P*
OS (fixed‐effects)	13	3.02 (2.35–3.89)	< 0.01*	< 0.01*	22.40	0.22
Tumor type						
Osteosarcoma	10	3.15 (2.39–4.14)	< 0.01*	< 0.01*	21.30	0.25
Nonosteosarcoma	3	2.38 (1.24–4.58)	0.01*	0.01*	41.6	0.18
Pretherapy (fixed‐effects)	11	2.96 (2.28–3.84)	< 0.01*	< 0.01*	26.90	0.19
Y	7	2.56 (1.81–3.62)	< 0.01*	< 0.01*	0.00	1.00
*N*	4	3.59 (2.40–5.35)	< 0.01*	< 0.01*	73.80	0.01
MFS (random‐effects)	5	5.22 (2.08–13.08)	< 0.01*	< 0.01*	78.30	< 0.01
Sample source						
Asian	3	8.93 (3.30–24.15)	< 0.01*	< 0.01*	53.40	0.12
Non‐Asian	2	2.18 (1.13–4.20)	0.02*	0.02*	30.10	0.23
Sample size						
*n* ≥ 70	2	2.41 (1.12–5.21)	0.03*	0.03*	54.50	0.14
*n* < 70	3	9.23 (3.38–25.24)	< 0.01*	< 0.01*	46.90	0.15
Analysis model						
Univariate	2	4.14 (0.75–22.99)	0.10	0.10	91.50	< 0.01
Multivariate	3	6.21 (2.13–18.13)	< 0.01*	< 0.01*	49.90	0.14
Publication date						
> 2010	2	2.18 (1.13–4.20)	0.02*	0.02*	30.10	0.23
≤ 2010	3	8.93 (3.30–24.15)	< 0.01*	< 0.01*	53.40	0.12
Tumor type						
Osteosarcoma	2	10.18 (1.19–87.05)	0.03*	0.03*	70.90	0.06
Nonosteosarcoma	3	4.04 (1.35–12.12)	0.01*	0.02*	83.80	< 0.01
EFS (fixed‐effects)	4	1.07 (1.03–1.11)	< 0.01*	< 0.01*	38.90	0.18
Tumor type						
Osteosarcoma (random‐effects)	3	1.20 (0.74–1.96)	0.46	1.38	59.10	0.09
Nonosteosarcoma	1	1.00 (0.35–2.87)	1.00	1.00	–	–
DSS	1	4.54 (2.92–40.89)	0.03*	0.09	–	–

* Statistically significant.

### Correlation between ezrin expression and clinicopathological outcomes

To elucidate the clinicopathological significance of ezrin expression, comprehensive meta‐analyses were conducted to evaluate the correlation between ezrin expression and CP that also considered patient age and gender, tumor size, location, grade and stage, metastasis, recurrence, and chemotherapy response (CR). As obvious heterogeneity was observed in the analysis of metastasis (*I* ^2^ = 67.4% *P* < 0.01) and tumor grade (*I* ^2^ = 66.00% *P* = 0.01), a random‐effects model was used for each analysis. A fixed‐effects model was used for each of the other analyses. As was the case for the analyses of survival outcomes, subgroup analyses according to tumor type (osteosarcoma vs. nonosteosarcoma) were performed to evaluate the correlation between ezrin expression and CP. The statistical results showed that ezrin overexpression was positively correlated with higher rates of tumor metastasis (OR 6.59, 95% CI: 2.84–15.33, *P* < 0.01, *P*_FDR_ < 0.01) and recurrence (OR 3.18, 95% CI: 1.88–5.37, *P* < 0.01, *P*_FDR_ < 0.01) and more advanced tumor grade (OR 3.252, 95% CI: 1.371–7.715, *P* = 0.01, *P*_FDR_ = 0.03), which was specifically correlated with osteosarcoma but not with other CP. The statistical analyses are summarized in Table 3.

**Table 3:** Summary of correlation between ezrin expression and CP.

Category	Study (*n*)	Heterogeneity		Effects model	OR (95% CI)	*P* value	*P*_FDR_
		*I^2^*	*P*				
Age	10	42.30	0.08	Fixed	1.21 (0.87–1.69)	0.26	0.33
Nonosteosarcoma	4	60.40	0.06	Random	0.94 (0.41–2.18)	0.89	0.89
Osteosarcoma	6	29.40	0.22	Fixed	1.40 (0.90–2.20)	0.14	0.21
Gender	12	0.00	0.87	Fixed	0.89 (0.66–1.20)	0.45	0.50
Nonosteosarcoma	5	0.00	0.53	Fixed	0.94 (0.60–1.46)	0.77	0.81
Osteosarcoma	7	0.00	0.83	Fixed	0.86 (0.57–1.28)	0.45	0.50
Tumor size	7	16.40	0.31	Fixed	1.24 (0.86–1.78)	0.25	0.33
Nonosteosarcoma	5	39.20	0.16	Fixed	1.07 (0.61–1.88)	0.80	0.82
Osteosarcoma	2	0.00	0.83	Fixed	1.65 (0.71–3.82)	0.24	0.33
Tumor localization	12	0.00	0.74	Fixed	0.84 (0.58–1.23)	0.37	0.44
Nonosteosarcoma	5	0.00	0.41	Fixed	0.68 (0.41–1.12)	0.12	0.21
Osteosarcoma	7	0.00	0.90	Fixed	1.13 (0.64–1.99)	0.68	0.74
Tumor grade	6	66.00	0.01	Random	3.25 (1.37–7.72)	0.01*	0.03*
Sample source							
Asian	4	48.00	0.12		8.46 (3.40–21.09)	< 0.01*	< 0.01*
Non‐Asian	2	0.00	0.66		1.90 (0.83–4.35)	0.13	0.21
Publication date							
≥ 2011	3	85.00	< 0.01		3.84 (0.69–21.46)	0.13	0.21
< 2011	3	0.00	0.53		2.86 (1.37–5.96)	0.01*	0.03*
Sample size							
**< **60	3	39.90	0.19		4.56 (1.29–16.13)	0.02*	0.05
≥ 60	3	80.30	0.01		2.60 (0.75–9.00)	0.13	0.21
Tumor type							
Nonosteosarcoma	4	70.90	0.02		2.35 (0.90–6.16)	0.08	0.16
Osteosarcoma	2	0.00	0.71		9.55 (2.55–35.82)	< 0.01*	< 0.01*
Tumor stage	7	0.00	0.47	Fixed	1.69 (1.03–2.78)	0.04*	0.10
Nonosteosarcoma	3	33.00	0.23	Fixed	1.69 (0.84–3.39)	0.14	0.21
Osteosarcoma	4	0.00	0.46	Fixed	1.70 (0.84–3.42)	0.14	0.21
Metastasis	11	67.40	< 0.01	Random	6.59 (2.84–15.33)	< 0.01*	< 0.01*
Sample source							
Asian	7	44.60	0.09		14.26 (5.74–35.45)	< 0.01*	< 0.01*
Non‐Asian	4	46.10	0.14		1.93 (0.77–4.85)	0.16	0.23
Publication date							
≥ 2010	6	68.20	0.01		3.75 (1.28–11.03)	0.02*	0.05
< 2010	5	54.70	0.07		13.56 (4.12–44.66)	< 0.01*	< 0.01*
Sample size							
< 55	6	44.3	0.11		5.11 (2.24–11.67)	< 0.01*	< 0.01*
≥ 55	5	81.8	< 0.01		10.46 (1.66–65.75)	0.01*	0.03*
Tumor type							
Nonosteosarcoma	3	73.2	0.02		4.17 (0.92–18.84)	0.06	0.13
Osteosarcoma	8	68.4	< 0.01		8.36 (2.82–24.76)	< 0.01*	< 0.01*
Recurrence	6	46.5	0.10	Fixed	3.18 (1.88–5.37)	< 0.01*	< 0.01*
Nonosteosarcoma	3	63.5	0.07	Random	3.29 (0.95–11.40)	0.06	0.13
Osteosarcoma	3	47.7	0.15	Fixed	2.95 (1.32–6.58)	0.01*	0.03*
CR	4	28.9	0.24	Fixed	1.28 (0.77–2.13)	0.35	0.43

* Statistically significant.

As obvious heterogeneity was observed in the analyses of tumor grade and metastasis, subgroup analyses stratified according to sample source, publication date, sample size, and tumor type were conducted. The results showed that the overall heterogeneity was not effectively reduced and that the sample source might be the underlying source of heterogeneity (Table 3).

### Publication bias and sensitivity analysis

Funnel plot analysis (Fig. 3) and Begg's and Egger's tests (Table 4) were used to assess the publication bias. For the analysis of tumor stage, there was no consensus regarding the presence of publication bias. For the analysis of tumor metastasis, an obvious publication bias was observed. A trim‐and‐fill analysis was performed for each analysis. The results showed that no additional studies were needed to reduce the publication bias for the tumor stage analysis (Fig. 4A). However, three more studies, which might have been reports of negative results, were needed to reduce the publication bias for the tumor metastasis analysis (Fig. 4B). For each of the other prognostic and CP, no obvious publication bias was observed (Table 4).

**Figure 3:** Funnel plots for OS (A), MFS (B), EFS (C), and patient age and gender, tumor size and localization, grade and stage, metastasis, recurrence, and CR (D–L, respectively).

**Table 4:** Begg’s test and Egger’s test for publication bias.

Analysis value	Study (*n*)	Begg’s test		Egger's test	
		*z*	*P*	*t*	*P*
OS	13	0.06	0.95	0.00	1.00
MFS	5	0.24	0.81	2.73	0.07
EFS	4	0.34	0.73	0.42	0.72
Age	10	0.72	0.47	0.01	0.99
Gender	12	0.34	0.73	0.11	0.92
Tumor size	7	1.20	0.23	−0.90	0.41
Tumor localization	12	0.89	0.37	0.47	0.65
Tumor grade	6	0.75	0.45	1.51	0.21
Tumor stage	7	2.10	0.04*	2.56	0.05
Metastasis	11	2.18	0.029*	3.13	0.012*
Recurrence	6	0.00	1.000	0.54	0.615
CR	4	0.34	0.734	−0.26	0.820

* Significant difference.

**Figure 4:** Trim‐and‐fill analysis for tumor stage (A) and metastasis (B). Dot, included studies; square, filled studies.

Sensitivity analysis was performed to assess the stability of our results. In the sensitivity analysis for OS, the results showed that one study 31 might influence the stability of the analysis (Fig. 5A). The results were stable when this study was omitted (Fig. 5B), and the significance of the association of ezrin expression and OS was not altered (HR 2.582 95% CI: 1.940–3.437, *P* < 0.01, *P*_FDR_ < 0.01); in addition, no obvious heterogeneity was observed (*I* ^2^ = 0.00% *P* = 0.52). Sensitivity analyses for EFS and CR were not performed because a limited number of studies were included (*n* < 5). The sensitivity analyses for MFS and CP showed that our results were stable (Figs 5C,D–K).

**Figure 5:** Sensitivity analysis for OS (A), OS omitting one study (B), MFS (C), and patient age and gender, tumor size and localization, grade and stage, metastasis, and recurrence (D–K, respectively).

## Discussion

Ezrin is a member of the evolutionarily conserved ERM protein family, which contains proteins involved in cellular structure that act as cytoskeletal linkers. By coupling transmembrane proteins to the actin cytoskeleton or modulating cellular signal transduction, ezrin plays a role in cancer progression involving cancer cell adhesion, migration, growth, and metastasis 9, 10, 11, 12. In 2007, Bruce et al. 40 conducted a large‐scale study to explore ezrin expression in various cancers using microarray IHC. The results suggested that ezrin expression is significantly increased in cancers of mesenchymal origin (sarcomas). The prognostic value of ezrin has been proposed for numerous types of cancers 13, 14, 15, 16. However, the clinical prognostic significance of ezrin in patients with bone and soft tissue sarcomas remains inconclusive.

Previously, a meta‐analysis was conducted to evaluate the prognostic value of high ezrin expression in patients with solid tumors, including bone and soft tissue sarcomas 20; however, the number of included studies was limited (*n* = 9), and therefore, the results were inconclusive. In the present study, 19 studies with a total of 1316 bone and soft tissue sarcoma patients were included to evaluate the clinicopathological and prognostic value of ezrin expression. The results showed that positive/high ezrin expression was significantly associated with poor prognosis in patients with bone and soft tissue sarcomas, which was consistent with the results of previous analyses in patients with solid cancers 20. Moreover, subgroup analysis according to tumor type showed that ezrin overexpression could predict poor OS and MFS in both osteosarcoma and nonosteosarcoma, even though most of the data were from patients with osteosarcoma. As chemo/radiotherapy was of great importance to patient prognosis, a stratified analysis of the effect of prechemotherapy/radiotherapy on OS was conducted, and the results showed that the prognostic value of ezrin expression in patients with bone and soft tissue sarcomas was not altered. Moreover, the overall effects were not altered in the subgroup analyses, suggesting that the results of the present study are credible. In addition, no publication bias was observed for the analyses of survival outcomes, and the results of the sensitivity analyses showed that our analyses were robust.

Regarding the correlation between ezrin expression and CP, the results of the pooled data analysis showed that ezrin overexpression was significantly correlated with an increased rate of tumor metastasis and recurrence, which was specifically notable for osteosarcoma. This was consistent with the results of a previous meta‐analysis in patients with osteosarcoma 41 and might have been caused by the limited number of studies of nonosteosarcoma that were included. In a recent meta‐analysis 42, the results showed that ezrin expression was not correlated with the distant metastasis of either gastric or esophageal cancers. Ezrin was suggested to be involved in the metastasis of osteosarcoma 43, 44, and the underlying molecular mechanism involved in the modulation of metastasis by ezrin might be different in different cancers. Previous studies showed that a significant change in ezrin expression was correlated with tumor responses to chemotherapy 45, 46. The results of the present study showed that ezrin expression was not correlated with tumor responses to chemotherapy. Although the underlying mechanisms involved in the effects of ezrin on the progression of bone and soft tissue sarcomas remain unclear and need further investigation, the results of our analysis showed that ezrin overexpression was significantly correlated with more advanced progression in patients with bone and soft tissue sarcomas, which might contribute to the strengths of the survival meta‐analysis.

Moreover, as obvious heterogeneity was observed in the analysis, random‐effects model and subgroup analyses were performed. Several characteristics of the patients and the studies, such as sample source, sample size, and publication date, might be underlying sources of heterogeneity in the meta‐analysis, and similar results were observed in our study. In addition, differences in the detection techniques, such as antibody selection and dilution and antigen retrieval methods, could explain the heterogeneity. Sample type might be another source of heterogeneity due to differences in the sampling methods used, such as tissue microarray (TMA) sampling, which may lead to more false‐negative results.

Several limitations of the present meta‐analysis should be considered. First, although the results showed there was no obvious publication bias, some other potential sources of publication bias should be taken into consideration, such as unpublished negative results 22 or studies that could not be included due to language limitations. Second, most of the HRs and the corresponding 95% CIs were extracted indirectly, and there was obvious uniformity in terms of the definitions of survival outcomes, which might have an impact on the reliability of our results. Third, different definitions of what is considered to be ezrin positive were observed in the studies, which might have been a result of differences in the detection methods and the definitions of the cutoff values and may have led to interstudy heterogeneity. In the present analysis, only studies using IHC‐based detection methods were included. Variations in the definitions of the cutoff values (staining scores or percentages of positive cells) might be due to the characteristics of certain sarcomas or authors’ preferences. Further study is needed to investigate whether the cutoff value could impact the prognostic value of ezrin for sarcomas, which remained vague due to the limited number of studies included and the lack of uniformity in terms of what was considered ezrin positive in the present analysis.

In addition, this meta‐analysis is a retrospective study, and most of the included studies investigated the clinical significance of ezrin expression in patients with osteosarcoma (12 of 19), which might lead to subject selection bias. Moreover, the recruitment of ezrin to areas of the plasma membrane is important for the functional regulation of ezrin 47, 48 and published results could not be used to reach a consensus 17, 25, and thus, the staining pattern or subcellular localization should be taken into consideration; however, insufficient data were extracted for analysis, and further investigation is needed.

## Conclusion

In the present meta‐analysis, the results showed that ezrin overexpression was significantly correlated with poor survival and more advanced tumor progression in patients with bone and soft tissue sarcomas, which suggested that ezrin is a valuable prognostic biomarker as well as a potential therapeutic target, although further comprehensive investigations with consistent methodologies are needed to validate our results.

## Conflict of interest

The authors declare no conflict of interest.

## Author contributions

FW and ZYZ conceived and designed the project and wrote the manuscript; FW, TY, and ZYZ analyzed and interpreted the data; and all authors participated in acquiring the data and have read and approved the final version of the manuscript.
